# miR-22 Suppresses EMT by Mediating Metabolic Reprogramming in Colorectal Cancer through Targeting MYC-Associated Factor X

**DOI:** 10.1155/2022/7843565

**Published:** 2022-08-25

**Authors:** Shusen Xia, Xianyan Wang, Yi Wu, Tong Zhou, Hongpeng Tian, Zuoliang Liu, Lifa Li, Zaihua Yan, Guangjun Zhang

**Affiliations:** ^1^The Second Department of General Surgery, The Affiliated Hospital of the North Sichuan Medical College, Nanchong, 637000 Sichuan, China; ^2^Institute of Hepatobiliary, Pancreatic and Intestinal Disease, The Affiliated Hospital of the North Sichuan Medical College, Nanchong, 637000 Sichuan, China; ^3^West China Hospital, Sichuan University-Ying Shan Hospital, Nanchong, 637000 Sichuan, China; ^4^The Pain Department, The Affiliated Hospital of the North Sichuan Medical College, Nanchong, 637000 Sichuan, China

## Abstract

Colorectal cancer (CRC) is one of the most frequent gastrointestinal cancers. MicroRNAs (miRNAs) have been proved to be unusually expressed in CRC progression and thus alter multiple pathological processes in CRC cells. However, the specific roles and mechanisms of miR-22 in CRC have not been clearly reported. MicroRNA-22 (miR-22) and MYC-associated factor X (MAX) expressions were determined by RT-qPCR in CRC tissues and cells. The targeted regulatory effects of miR-22 and MAX were confirmed by luciferase reporter and coimmunoprecipitation assays. Also, gain- and loss-of-function and rescue experiments were used to elucidate the function and mechanism of miR-22 and MAX in CRC cells and the mouse xenograft model. We discovered that miR-22 was hypermethylated and downregulated, while MAX was upregulated in CRC. miR-22 markedly inhibited migration, invasion, glycolysis, and cancer stem cell transcription factors in CRC cells. In addition, it was found that miR-22 can directly target MAX. Additional functional experiments confirmed that MAX overexpression can rescue the effects of miR-22 on the behavior of CRC cells. This study suggested that miR-22, as a cancer suppressor, participates in CRC progression by targeting MAX, which might provide basic information for therapeutic targets for CRC.

## 1. Introduction

Colorectal cancer (CRC) is one of the most common gastrointestinal cancers [1]. Globally, there are about 1.2 million new cases of CRC each year, and 600,000 people die from it [2]. Because early clinical symptoms of CRC patients are not obvious and there is a lack of effective diagnostic markers, the diagnostic rate of early CRC is low [3]. About 15-25% of CRC patients have liver metastases at diagnosis [4]. After surgery, radiotherapy, and chemotherapy, the clinical symptoms of most patients experience remission, but the 5-year survival rate is still low [5]. Therefore, prognostic markers of CRC are of great significance for early diagnosis. Research demonstrated that the application of different biomarkers can provide early diagnostic and prognostic direction for CRC, which also has a good improvement potential on the prognosis of CRC [6, 7]. However, the mechanisms in CRC lesions and progression are not fully understood. Therefore, it is of great theoretical and practical significance to confirm the relevant mechanisms of CRC and screen new specific biomarkers and targeted drugs for the diagnosis, treatment, and prognosis of CRC patients.

The epigenetic information of the genome is that the DNA sequence is unchanged, but the phenotype is altered, and this phenotypic alteration can be stably inherited during development and cell proliferation [8]. DNA methylation is a hot spot of epigenetic tumor research, which is mainly located in the CpG island of genes [9]. Abnormal methylation of gene promoters is one of the most frequent mechanisms of inactivation of tumor suppressors and other genes [10]. Therefore, the methylation level of certain genes can be an effective biomarker to assess the prognosis, recurrence, and early diagnosis of patients and even become therapeutic targets. Research showed that DNA methylation and miRNAs have mutual regulation and mutual targeting effects [11, 12]. The promoter regions of some miRNAs have CpG islands, and abnormal hypermethylation can cause their low expression, leading to tumorigenesis [13]. There have also been reports that miRNAs can result in abnormal changes in DNA methylation by targeting DNMT1 and DNMT3 [14]. Therefore, the regulatory relationship between DNA methylation and miRNAs is of great significance for the in-depth understanding of the network regulation mechanism of gene expression.

MicroRNAs (miRNAs), as noncoding RNAs, can regulate gene expression by targeting the binding sites of mRNAs, thereby affecting multiple biological processes including immune system activation, inflammatory response, cholesterol homeostasis, and glycolysis [15–18]. miRNAs can also participate in tumor biological processes, including cell growth, differentiation, and apoptosis [15, 19]. Due to genetic polymorphism, expression of miRNAs and their stability in body fluids show that miRNAs can be applied as markers for clinical diagnosis and prediction of tumors, as well as to assess the invasion, metastasis, and sensitivity to chemotherapeutic drugs of CRC [20]. It was reported that miR-22, as a tumor suppressor, plays a key role in colorectal cancer, liver cancer, and other diseases [21, 22]. For example, miR-22 suppresses lung cancer by inhibiting cell growth via the MET/STAT3 pathway [23]. We also discovered by biological prediction that miR-22 is located near the CpG island, suggesting that epigenetic regulation may participate in CRC progression as an upstream regulatory mechanism of miR-22. However, the specific mechanism of miR-22 in colorectal cancer is still unclear.

MYC-associated factor X (MAX) is a member of the bHLHLZ (basic helix-loop-helix leucine zipper) family, and MAX functions as a transcription factor by forming a dimer with MYC, resulting in promoting or inhibiting the transcription and expression of MYC targets [24]. In our study, we proposed for the first time that as a key link in CRC, the upstream of miR-22 can be regulated by epigenetic DNA methylation. Then, we investigated expression changes and methylation of miR-22 in CRC tissues and confirmed the influences of miR-22 overexpression or knockdown on biological functions in CRC cells and the mouse model. Most importantly, the possible regulatory mechanism of miR-22 in CRC progression was explored. The clarification of the above questions will enable further clarification of the mechanism of miR-22 in the CRC process and provide a theoretical basis for the possibility of miR-22 as a new therapeutic target of CRC.

## 2. Materials and Methods

### 2.1. Patients and Samples

CRC and paracarcinoma tissues were harvested from 20 CRC patients, who were admitted to the Affiliated Hospital of the North Sichuan Medical College between 2018 and 2019. The patients were informed and signed the informed consent. The ethical approval for this study was obtained from the Ethics Committee of the Affiliated Hospital of the North Sichuan Medical College (Approval No. 2021ERCA7005). After resection, all samples were immediately placed in liquid nitrogen. None of the patients had received surgery on the same site or had disease in other hospitals before treatment and had no history of radiotherapy or chemotherapy.

### 2.2. Cell Culture

Normal human fetal colon (FHC; CRL-1831), SW620 (CCL-227), LoVo (CCL-229), HCT116 (CCL-247), SW480 (CCL-228), and HT29 (HTB-38) cells were from ATCC. FHC cells were grown in DMEM: F12 medium (Life Technologies; 11330057); SW620 and SW480 cells were grown in L-15 medium (Gibco, 11415); LoVo cells were grown in F12K medium (Invitrogen); HCT116 cells were grown in DMEM (Gibco); and HT29 cells were grown in McCOY's 5A (Sigma; M4892). All media received 10% fetal bovine serum (FBS, Sigma) and penicillin/streptomycin. All cells were cultured at 37°C and 5% CO_2_.

### 2.3. Cell Transfection

miR-22 mimics, inhibitors, and negative control (NC) were purchased from GenePharma (Suzhou, China). MAX-overexpressed plasmids were established through amplification of MAX full-length cDNAs and cloning of gene products into the pcDNA 3.1 vector, and the sequencing was confirmed. In brief, SW620 and HCT116 cells were transfected with oligonucleotides and plasmids using Lipofectamine 3000 (Invitrogen) for 48 h. In the rescue experiment, miR-22 mimic and MAX-overexpressed plasmids were cotransfected.

### 2.4. Bisulfite Sequencing PCR (BSP)

In line with the literature [25], the methylation level of miR-22 was confirmed using the BSP method. Briefly, genomic DNA was extracted using standard protease K digestion and phenol/chloroform methods. The extracted genomic DNA was modified with bisulfite. The modification consisted of alkaline denaturation, vulcanization, dehydrogenation, purification, desulfurization, sedimentation, and recovery. The bisulfite-treated DNA was used as a template for PCR amplification. PCR products were purified using a gel purification kit (Qiagen), cloned into pMD18-T vectors (Takara) to construct plasmids, and then sequenced.

### 2.5. RT-qPCR

We extracted total RNAs by applying TRIzol reagent (Invitrogen, MA, USA). Then, the extracted RNA samples were reversed-transcribed into cDNAs using the PrimeScript™ RT Reagent Kit (Takara). Expressions of genes were monitored by the SYBR Green qPCR master Mix (DBI Bioscience). The data were calculated with the 2^-*ΔΔ*Ct^ method.

### 2.6. Western Blot

Total proteins were extracted after cell lysis with the RIPA lysis buffer (Beyotime, China). After quantification, 40 *μ*g protein was subjected to electrophoresis and transferred onto PVDF membranes. After blocking, the membranes were exposed to specific primary antibodies at 4°C overnight and secondary antibodies for 2 h. The results were visualized with the chemiluminescent reagent (Millipore, Burlington, MA, USA). The quantification of Western blot bands was performed using ImageJ software (Bethesda, Maryland, USA).

### 2.7. Transwell Assay

Chamber inserts (Corning Inc.) were precoated with diluted Matrigel (0.3 mg/mL; BD Biosciences) for 30 min at 37°C. Then, the transfected CRC cells (5 × 10^5^ cells/well) in serum-free media were evenly placed into the upper chamber, and the medium supplemented with 20% FBS was placed in the lower chamber. After 24 h of incubation, the invaded cells were fixed and stained with 4% formaldehyde and 0.2% crystal violet, respectively. The invasive cells were recorded under a microscope.

### 2.8. Wound Healing

Transfected CRC cells (1 × 10^6^ cells/well) were inoculated in a 24-well plate at 37°C for 18 h. Scratches were made using a 100 *μ*L pipette tip. After washing, the images were captured.

### 2.9. Detection of Glucose Consumption, ATP, and Lactic Acid

According to the instruction of the corresponding kits, the levels of glucose consumption, ATP, and lactic acid were examined using the glucose uptake colorimetric assay kit (Sigma-Aldrich, MAK083), the ATP assay kit (Abnova; KA1661), and the lactic acid assay kit (Sigma; MAK064-1KT), respectively.

### 2.10. Luciferase Reporter Assay

Wild-type (WT) and mutant (Mut) MAX plasmids were constructed by the pGL3-Basic vector in line with the predicted binding sites between the miR-22 and MAX promoter region. Next, SW620 cells were cotransfected with miR-22 mimics and pGL3-WT-MAX or pGL3-MUT-MAX for 48 h. The luciferase activity was assessed with the dual luciferase assay kit (Promega).

### 2.11. Coimmunoprecipitation (CO-IP) Assay

On the basis of previous studies [26, 27], the CO-IP assay was used to analyze the binding between miR-22 and MAX in CRC.

### 2.12. Tumor Xenograft Model

BALB/c nude mice (4-week-old, weighing 18-25 g) were from the Shanghai Laboratory Animal Center (Shanghai, China). All mice were raised in a sterile environment. SW620 cells were collected and counted, and 2 × 10^6^ cells/mL were injected into the right hind leg of the mice. The length and width of the tumors were monitored, and the tumor volume (formula: length × width2/2) was determined at 7, 14, 21, and 28 days. During this period, miR-22 was intravenously injected into the mice. After 28 days, the xenograft tumors in each group were obtained for subsequent analysis. This animal experiment was strictly conducted according to the Institutional Animal Protection and Use Committee.

### 2.13. H&E Staining

Referring to previous research [28], subcutaneous grafts of CRC cells in mice were fixed with 10% formaldehyde solution. The tissues were dehydrated, became transparent, and embedded after paraffin impregnation. The tissues were cut into 5 *μ*m slices and spread on glass slides with polylysine. After hematoxylin staining, dehydration, eosin staining, dehydration, xylene transparency, and neutral gum fixation, the pathological features were observed under a light microscope.

### 2.14. Statistical Analysis

Data are presented as the mean ± SD. SPSS 20.0 software (SPSS, Inc.) was used for data analysis with Student's *t*-test or one-way ANOVA. *P* < 0.05 indicates a statistical difference. All the experiments were performed at least three times.

## 3. Results

### 3.1. miR-22 Was Prominently Hypermethylated and Downregulated in CRC Tissues

The CpG island, as a key part of epigenetic regulation, is of crucial importance in gene regulation. To investigate the methylation state of miR-22 in CRC, we first predicted the CpG islands in the miR-22 promoter sequences through MethPrimer (Figure 1(a)). BSP results showed that miR-22 was methylated in both CRC and paracarcinoma tissues, while the methylation level of the miR-22 promoter was more prominent in CRC tissues than in paracarcinoma tissues (Figure 1(b)). In addition, RT-qPCR data certified that with respect to paracarcinoma tissues, miR-22 expression was prominently lowered in CRC tissues (Figure 1(c)). We also identified the associations between miR-22 and clinical features. The data indicated that a low miR-22 expression level was associated with poor prognostic markers, including distant metastases (*P* = 0.0248) and TNM stage (*P* = 0.0104), while no association was found for age, gender, and tumor size (Table 1). These findings showed that miR-22 is hypermethylated, while lowly expressed in CRC tissues, and miR-22 might be a potential predictor of metastatic recurrence in human CRC patients.

### 3.2. miR-22 Markedly Downregulated SOX2 and OCT4 in CRC Cells

To further demonstrate the action of miR-22 in CRC cells, first, the expression changes of miR-22 in different CRC cells were determined. As exhibited in Figure 2(a), miR-22 expression was markedly reduced in CRC cells relative to that in FHC cells (*P* < 0.05), and thus, CRC cells were used in subsequent experiments. Then, the miR-22 mimic and inhibitor were transfected into CRC cells. RT-qPCR results showed that relative to the NC group, miR-22 expression was notably upregulated in the mimic group, while it was markedly downregulated in the inhibitor group, indicating the successful overexpression and suppression of miR-22 in CRC cells (*P* < 0.05, *P* < 0.01, Figure 2(b)). Additionally, the data signified that overexpression of miR-22 markedly downregulated SOX2 and OCT4, and blockage of miR-22 upregulated SOX2 and OCT4 in CRC cells (Figure 2(c)). On the whole, it was found that aberrant expression of miR-22 is relevant to cancer stem cell transcription factors (SOX2 and OCT4) in CRC cells.

### 3.3. miR-22 Markedly Suppressed Migration and Invasion of CRC Cells

After overexpression or blockage of miR-22 in CRC cells, the influences of miR-22 on the migration and invasion of CRC cells were further verified. Transwell results showed that compared to the NC group, the number of invaded cells was decreased in the mimic group, while they were markedly increased in the inhibitor group, suggesting that overexpression of miR-22 prevents the invasion of CRC cells, and blockage of miR-22 accelerates the invasion of CRC cells (Figure 3(a)). Similarly, wound healing results signified that compared with the NC group, the migration index was markedly reduced in the mimic group, while it was elevated in the inhibitor group, indicating that overexpression of miR-22 suppresses the migration of CRC cells, and suppression of miR-22 facilitates the migration of CRC cells (Figure 3(b)). It was also discovered that overexpression of miR-22 raised E-cadherin and downregulated N-cadherin and Vimentin, and blockage of miR-22 lowered E-cadherin and upregulated N-cadherin and Vimentin in CRC cells (Figure 3(c)). In general, it was shown that miR-22 has a prominent inhibitory effect on the migration and invasion of CRC cells.

### 3.4. miR-22 Markedly Inhibited Glycolysis in CRC Cells

Aerobic glycolysis, as the hallmark of cancer cells, tends to rely on the aerobic glycolysis of glucose for energy. Therefore, we further determined whether miR-22 could alter the glycolysis of CRC cells. First, the results showed that overexpression of miR-22 markedly reduced glucose consumption, and blockage of miR-22 increased glucose consumption in CRC cells (Figure 4(a)). Second, it was discovered that overexpression of miR-22 markedly decreased the level of ATP, and blockage of miR-22 increased the level of ATP in CRC cells (Figure 4(b)). Third, the data showed that overexpression of miR-22 elevated the lactic acid level, and suppression of miR-22 lowered the lactic acid level in CRC cells (Figure 4(c)). Moreover, the data showed that overexpression of miR-22 markedly downregulated HK2, PKM2, and LDHA, and blockage of miR-22 markedly upregulated HK2, PKM2, and LDHA in CRC cells (Figure 4(d)). In short, we found that miR-22 has a significant weakening role on glycolysis in CRC cells.

### 3.5. miR-22 Specifically Downregulated MAX, Which Was Highly Expressed in CRC Tissues

Subsequently, we discovered through bioinformatics software predictions that there were underlying binding sites between miR-22 and MAX (Figure 5(a)). Luciferase reporter assay further verified that miR-22 overexpression could markedly reduce the luciferase activity of WT-MAX, indicating the targeted regulation of miR-22 on MAX (Figure 5(b)). Additionally, CO-IP results further proved the targeted regulation of miR-22 to MAX (Figure 5(c)). Western blot data showed that overexpression of miR-22 downregulated MAX, and blockage of miR-22 upregulated MAX in CRC cells (Figure 5(d)). In addition, RT-qPCR results showed that the level of MAX was markedly elevated in CRC tissues versus paracarcinoma tissues (Figure 5(e)). IHC data from online database, the Human Protein Atlas (https://www.proteinatlas.org/), and Western blot results showed that the expression trend of MAX in CRC tissues was consistent with RT-qPCR results (Figures 5(f) and 5(g)). We also discovered that there was a significant negative correlation between miR-22 and MAX in 40 CRC tissues (Figure 5(h)). In summary, our data showed that MAX, as a target gene of miR-22, is upregulated in CRC tissues.

### 3.6. Cotransfection Verification of miR-22 Mimic and MAX-Overexpressed Plasmids in CRC Cells

Based on the result that MAX, as a target gene of miR-22, could be distinctly downregulated by miR-22 in CRC, we further explored the impacts of miR-22 and MAX on the biological functions of CRC cells through rescue experiments. CRC cells were alone or cotransfected with miR-22 mimic and MAX-overexpressed plasmids. RT-qPCR data showed that miR-22 was upregulated, MAX was markedly downregulated in the mimic group relative to that in the NC group, MAX was markedly upregulated in the MAX-overexpressed group with respect to that in the vector group, miR-22 was markedly upregulated in the MAX overexpression+mimic group versus that in the MAX overexpression group, and MAX was markedly upregulated in the MAX overexpression+mimic group compared with that in the mimic group (Figures 6(a) and 6(b)). Western blot showed that overexpression of miR-22 notably reduced MAX expression, overexpression of MAX prominently elevated MAX expression, and overexpression of MAX o could also increase MAX expression, which was inhibited by the miR-22 mimic in CRC cells (Figure 6(c)). To sum up, we found that miR-22 mimic and MAX-overexpressed plasmids were successfully managed into CRC cells.

### 3.7. miR-22 Prominently Prevented the Migration and Invasion of CRC Cells through MAX

After successful cotransfection, we further determined the influences of miR-22 and MAX on the migration and invasion of CRC cells. Western blotting data showed that overexpression of miR-22 markedly upregulated E-cadherin and downregulated N-cadherin and vimentin in CRC cells, while the changes in these proteins mediated by miR-22 overexpression could be reversed by MAX overexpression (Figure 7(a)). Similarly, wound healing results showed that overexpression of MAX could promote cell migration in miR-22-overexpressed CRC cells (Figure 7(b)). Overexpression of MAX could also accelerate cell invasion in miR-22-overexpressed CRC cells (Figure 7(c)). Overall, these results showed that MAX is required for miR-22 to prevent the migration and invasion of CRC cells.

### 3.8. miR-22 Notably Prevented Glycolysis by Targeting MAX in CRC Cells

We also determined the impacts of miR-22 and MAX on the glycolysis and cancer stem cell transcription factors in CRC cells. First, it was found that overexpression of MAX could markedly increase glucose consumption, which was reduced by the miR-22 mimic in CRC cells, indicating that miR-22 overexpression notably attenuated glucose consumption induced by MAX in CRC cells (Figure 8(a)). Second, the data showed that overexpression of MAX could markedly reverse the increase of ATP mediated by the miR-22 mimic in CRC cells (Figure 8(b)). Third, the reduction of the lactic acid level mediated by miR-22 overexpression also could be notably weakened by MAX overexpression in CRC cells (Figure 8(c)). Western blotting data showed that overexpression of MAX could also notably upregulate SOX2 and OCT4, which were downregulated by the miR-22 mimic in CRC cells (Figure 8(d)). Furthermore, it was discovered that miR-22 overexpression markedly downregulated HK2, PKM2, and LDHA in CRC cells, while the changes in these proteins could be markedly attenuated by MAX overexpression (Figures 8(e) and 8(f)). As a whole, these data showed that MAX is also required for miR-22 to attenuate glycolysis and cancer stem cell transcription factors in CRC cells.

### 3.9. miR-22 Markedly Reduced Tumor Growth and Improved the Pathological Structure in the Mouse Xenograft Model of CRC

In line with the above findings *in vitro*, we speculated that miR-22 could also prevent tumor growth of CRC *in vivo*. To test this hypothesis, we established a xenograft mouse model through NC or miR-22 mimic-transfected SW620 cells to generate subcutaneous tumors. The data showed that the size of the tumors was prominently reduced after miR-22 overexpression after 28 days (Figures 9(a) and 9(b)). Also, the time-dependent analysis found that the volume of the tumors was remarkably inhibited in mice injected with the miR-22 mimic addressed SW620 cells relative to that of the NC group (Figure 9(c)). The weight of mice was also lower in the mimic group than that in the NC group (Figure 9(d)). In addition, H&E staining results showed that in blank and NC groups, there were a large number of necrotic cells with nuclear fragmentation and pyknosis, while the introduction of the miR-22 mimic could notably improve this pathological structure in the tumors of mice (Figure 9(e)). In summary, we proved that miR-22 can also block tumor growth and improve the pathological structure of CRC *in vivo*.

### 3.10. miR-22 Markedly Reduced MAX, SOX2, OCT4, and Glycolysis in the Mouse Xenograft Model of CRC

We further explored the impacts of miR-22 on MAX, SOX2, OCT4, and glycolysis *in vivo*. RT-qPCR data first found that MAX expression was markedly lowered, while miR-22 expression was markedly elevated in the miR-22-overexpression group versus that in the NC group (Figures 10(a) and 10(b)). Data also showed that overexpression of miR-22 could markedly downregulate MAX in CRC tumors (Figure 10(c)). As expected, E-cadherin was notably upregulated, and N-cadherin and Vimentin were prominently downregulated in the miR-22-overexpressed group versus the NC group (Figure 10(d)). Overexpression of miR-22 could also markedly reduce SOX2 and OCT4 in CRC tumors (Figure 10(e)). Furthermore, HK2, PKM2, and LDHA expressions were also inhibited by miR-22 overexpression *in vivo* (Figure 10(f)). Overall, our data showed that miR-22 can suppress MAX, SOX2, OCT4, and glycolysis *in vivo*.

## 4. Discussion

CRC is characterized by high morbidity and mortality and poor prognosis [7]. Recurrence and metastasis are the major causes of death in CRC patients, and prompt treatment can improve the survival of patients with nonmetastatic CRC [29]. Therefore, an in-depth understanding of the molecular pathways of CRC metastasis and the development of new prognostic molecular markers are helpful to reduce the occurrence of CRC metastasis. Studies found that miRNAs play key regulatory roles in multiple physiological processes, including cell migration, proliferation, differentiation, and apoptosis [18, 30, 31]. Various miRNAs are markers for predicting the prognosis of CRC [32, 33]. We further validated that miR-22 is distinctly downregulated in CRC, and miR-22 overexpression can also markedly prevent the metastasis of CRC cells. As reported in the literatures, miR-22 is associated with the suppression of CRC metastasis. For instance, miR-22 can notably restrain CRC invasion and metastasis through NLRP3 [34], miR-214 can also prominently suppress CRC cell metastasis by targeting BCL9L to inhibit the Wnt pathway [35], and miR-22 also has a blocking effect on the process of CRC metastasis by negative regulation of SP1 [36]. Therefore, our results are consistent with the results of previous studies. We further concluded that as a tumor suppressor gene, the dysfunction of miR-22 is likely to be one of the key reasons for accelerating the malignant progression of CRC.

Although miR-22 plays a crucial role in CRC metastasis, the mechanism of abnormal miR-22 expression in CRC is not fully understood. It was reported that DNA methylation and miRNA posttranscriptional regulation, as two key epigenetic regulatory mechanisms, have close regulatory relationships, and the revelation of their relationship is of great significance for further understanding the epigenetic regulation of disease-related gene expression [11]. It is of great value to apply miRNAs and disease-related DNA methylation status as molecular markers for diagnosis and prognosis, develop drugs specifically targeting DNA methylation and miRNAs, and develop new therapeutic methods for the related diseases [37]. Surprisingly, we predicted CpG islands in the miR-22 promoter sequences by MethPrimer. Our results also proved for the first time that miR-22 was markedly hypermethylated in CRC tissues, suggesting that the downregulation of miR-22 might be mediated by methylation in CRC.

Moreover, as reported in many studies [38, 39], miRNAs play a major role in the progression of malignant cancers. The dysfunction of miR-22 is also bound to cause the overimplementation of the downstream key protooncogenes in inducing the malignant behavior of cancer. Therefore, we further studied the key genes targeted by miR-22 in CRC. Through bioinformatics prediction, we accidentally found that miR-22 can potentially bind to the MAX promoter region, suggesting that MAX might be a targeted regulatory gene of miR-22. MAX is a universally expressed and highly conserved transcription factor, which is highly homologous to the primary structure of c-Myc. MAX can form heterodimers with c-Myc, Mad, or Mxil through its own bHLHZip domain and regulate the transcription of target genes, thus affecting cell proliferation, differentiation, or apoptosis [40, 41]. MYC has also been proven to be targeted and regulated by miR-22 to affect the progression of multiple cancers, including cervical cancer [42], acute myeloid leukemia [43], and gastric cancer [44]. Recent research also proved that MAX relates to cancer; for example, a decrease of MAX expression might be a latent marker of poor prognosis in anaplastic large cell lymphoma [24]. Therefore, we hypothesized that MAX is related to CRC progression, which could also be targeted by miR-22. Interestingly, it was discovered that miR-22 can directly target MAX, and MAX can reverse the blockage of miR-22 on the EMT, metastasis of CRC cells, indicating that MAX is involved in miR-22-mediated changes in CRC cell functions including metastasis.

More importantly, we further explored the effects of the miR-22/MAX axis on other functions of CRC in addition to metastasis. Stem cell-related molecules are a class of molecules that are specifically expressed in undifferentiated cells [45]. They are critical in maintaining the undifferentiated state of stem cells and regulating stem cell self-renewal [46]. One of the most striking features that stem cells and cancer cells have in common is their ability to self-renew. SOX2 and OCT4, as transcription factors, can sustain the phenotype of pluripotent embryonic stem cells [47]. Studies suggested that abnormal activation of SOX2 and OCT4-regulated networks can cause abnormalities of multiple signaling pathways and even form cascading amplifying effects [48, 49]. Through the verification of SOX2 and OCT4 expressions, we discovered that overexpression of miR-22 can reduce the levels of SOX2 and OCT4 through inhibiting MAX in CRC cells, indicating that the miR-22/MAX axis might downregulate SOX2 and OCT4 to affect the self-renewal ability of CRC cells.

The tumor microenvironment is also one of the most momentous factors in cancer, which is connected to energy metabolism [50]. Glucose metabolism, dominated by aerobic metabolism, is the main way for cells to obtain energy, while the process of transformation from normal cells to tumor cells is often accompanied by the remolding of metabolic pathways [51]. Cancer cells tend to rely on aerobic glycolysis of glucose for energy, whether or not there is sufficient oxygen around them [52]. The glycolysis rate of rapidly growing tumor cells is usually 200 times higher than that of cells in normal tissue [51]. The glycolytic pathway, as the initial stage of glucose utilization by cells, contains three key enzymes: HK, PFK, and PKM2 [53]. In our study, through the detection of indicators related to the glycolytic pathway, we also discovered for the first time that miR-22 can dramatically prevent glycolysis by MAX in CRC cells. In summary, miR-22 can not only suppress metastasis but also improve self-renewal and the glycolytic pathway of CRC cells by targeting MAX.

## 5. Conclusions

Our current study uncovered the following novel findings: (1) miR-22 is hypermethylated and downregulated in CRC tissues; (2) miR-22 is a functional tumor suppressor in CRC, which can suppress EMT, migration, invasion, and glycolysis of CRC cells; (3) miR-22 directly targets MAX in CRC; and (4) miR-22 can prevent CRC progression by targeting MAX (Figure 11). Therefore, the miR-22/MAX axis might provide an effective targeted therapy for CRC. This study did not address how the miR-22 promoter region is methylated, and this issue will be further explored in subsequent studies.

## Figures and Tables

**Figure 1:** miR-22 was markedly hypermethylated and downregulated in CRC tissues. (a) Bioinformatics prediction of the CPG island in miR-22 promoter regions. (b) The methylation status of miR-22 promoter regions was evaluated by the BSP method in CRC (*n* = 40) and paracarcinoma tissues (*n* = 40). (c) Expressions of miR-22 were confirmed using RT-qPCR assay in CRC (*n* = 40) and paracarcinoma tissues (*n* = 40).

**Figure 2:** miR-22 notably downregulated SOX2 and OCT4 in CRC cells. (a) Differential expression of miR-22 was assessed by RT-qPCR in normal human fetal colon (FHC) and 5 CRC cell lines (SW620, SW480, LoVo, HCT116, and HT29). (b) Verification of miR-22 overexpression and suppression was conducted through RT-qPCR in CRC cells. (c) After transfection with the miR-22 mimic or inhibitor, the protein levels of SOX2 and OCT4 were verified with Western blot in CRC cells.

**Figure 3:** miR-22 notably suppressed migration and invasion of CRC cells. CRC cells were transfected with the miR-22 mimic or inhibitor, respectively. (a) The invaded cells were determined by Transwell assay in miR-22-overexpressed or inhibited CRC cells. (b) Cell migration was assessed by wound healing in CRC cells after miR-22 overexpression or silencing, and the migration index was determined. (c) Western blot was conducted to identify expression changes of E-cadherin, N-cadherin, and Vimentin in miR-22-overexpressed or inhibited CRC cells.

**Figure 4:** miR-22 markedly inhibited glycolysis in CRC cells. CRC cells were transfected with the miR-22 mimic or inhibitor, respectively. (a) The quantity of glucose consumption was tested in miR-22-overexpressed or inhibited CRC cells. (b) The ATP kit was applied for the determination of the ATP level. (c) The lactic acid assay kit was used for the detection of the lactic acid level. (d) Western blotting analysis of HK2, PKM2, and LDHA in the managed CRC cells.

**Figure 5:** miR-22 specifically downregulated MAX, which was highly expression in CRC tissues. (a) The binding sites between miR-22 and MAX were predicted. (b) The direct targeting relationship of miR-22 and MAX was determined through the luciferase reporter assay. (c) The relationship of miR-22 and MAX was determined using CO-IP assay with the anti-Ago2 antibody. (d) The impacts of miR-22 overexpression or inhibitor on MAX expression were confirmed by Western blotting analysis in CRC cells. (e) Expression of MAX was determined through RT-qPCR in CRC (*n* = 40) and para-carcinoma tissues (*n* = 40). The expression change of MAX was also determined using IHC (online database results) (f) and Western blot assays (g). (h) The relevance between miR-22 and MAX was analyzed with Pearson correlation analysis in CRC tissues (*P* = 0.046). Para-T: paracarcinoma tissues; T: tumor tissues.

**Figure 6:** Cotransfection verification of miR-22 mimic and MAX-overexpressed plasmids in CRC cells. CRC cells were transfected with miR-22 mimic or/and MAX-overexpressed plasmids, respectively. The levels of miR-22 and MAX were determined by RT-qPCR analysis in SW620 (a) and HCT116 cells (b). Western blot was conducted to determine the protein level of MAX in the transfected CRC cells (c).

**Figure 7:** miR-22 markedly prevented the migration and invasion of CRC cells through MAX. miR-22 mimic and MAX-overexpressed plasmids that were individually or in combination transfected into CRC cells, respectively. (a) Identification of E-cadherin, N-cadherin, and Vimentin expressions through Western blotting analysis in each group. (b) Wound healing was used to monitor the cellular migration capacity in each group. (c) Transwell assay was used to examine the cellular invasion capacity in each group.

**Figure 8:** miR-22 notably prevented glycolysis by targeting MAX in CRC cells. CRC cells were transfected with miR-22 mimic and MAX-overexpressed plasmids alone or in combination, respectively. (a) Glucose consumption was determined in each group. (b) The ATP level was determined by the ATP kit in each group. (c) The level of lactic acid was determined by the lactic acid assay kit in each group. (d) Western blotting analysis of SOX2 and OCT4 in each group. (e) HK2, PKM2, and LDHA expressions were analyzed using Western blot in each group. (f) MAX and MYC expressions were evaluated by Western blotting analysis in each group.

**Figure 9:** miR-22 markedly reduced tumor growth and improved the pathological structure in the mouse xenograft model of CRC. SW620 cells (2 × 10^6^) transfected with the NC or miR-22 mimic were subcutaneously injected into nude mice, respectively. (a) Oncogenic mice are shown in each group. (b) Representative images of tumors are displayed in the mice implanted with NC or miR-22 mimic-transfected SW620 cells. (c) Changes in the tumor volume were determined on the 0, 7rd, 14th, 21th, and 28th days after subcutaneous injection. (d) Tumor weight was measured in each group. (e) The pathological structure of tumors in each group was assessed with H&E staining.

**Figure 10:** miR-22 markedly reduced MAX, SOX2, OCT4, and glycolysis in the mouse xenograft model of CRC. Nude mice were subcutaneously injected with NC or miR-22 mimic-managed SW620 cells, respectively. RT-qPCR analysis of MAX (a) and miR-22 (b) expressions in each group of tumors. (c) MAX expression was confirmed by Western blotting analysis in each group of tumors. (d) Validation of E-cadherin, N-cadherin, and Vimentin expressions through Western blotting analysis in each group of tumors. (e) Western blotting analysis of SOX2 and OCT4 in each group of tumors. (f) Western blot was used to monitor the expression changes of HK2, PKM2, and LDHA in each group of tumors.

**Figure 11:** Graphic abstract of this study.

**Table 1:** The correlation between clinical CRC patients' features and miR-22 expression.

Features	Numbers	miR-22 expression		*P* value
Gender		Low	High	
Female	18	8	10	0.7512
Male	22	12	10	
Age				
<50	21	13	8	0.2049
≥50	19	7	12	
Tumor size				
<4.5	27	11	16	0.176
≥4.5	13	9	4	
Distant metastases				
No	22	7	15	0.0248
Yes	18	13	5	
TNM stage				
I + II	21	6	15	0.0104
III + IV	19	14	5	

## Data Availability

The data generated during and/or analyzed during the current study are available from the corresponding author on reasonable request.
